# Aurantiamide Acetate Ameliorates Lung Inflammation in Lipopolysaccharide-Induced Acute Lung Injury in Mice

**DOI:** 10.1155/2022/3510423

**Published:** 2022-08-22

**Authors:** Zhengyu Fang, Jie Fang, Chunxiao Gao, Yueguo Wu, Wenying Yu

**Affiliations:** ^1^Key Laboratory of Neuropsychiatric Drug Research of Zhejiang Province, Hangzhou Medical College, Hangzhou, China; ^2^Zhejiang Provincial Laboratory of Experimental Animal's & Nonclinical Laboratory Studies, Hangzhou Medical College, Hangzhou, China

## Abstract

**Purpose:**

Aurantiamide acetate (AA) is a dipeptide derivative with complex pharmacological activities and remarkable effects on preventing and treating various diseases. In the current study, we aimed to investigate whether AA can exert protective effects in a mouse model of ALI induced by LPS.

**Materials and Methods:**

In this model, mice were given intranasal LPS for 3 days prior to receiving AA (2.5, 5, and 10 mg/kg) via oral gavage. An assessment of histopathological changes was performed by hematoxylin and eosin (HE). Proinflammatory cytokines were detected in bronchoalveolar lavage fluids (BALFs) by enzyme-linked immunosorbent assays (ELISAs). The effects of AA on protein expression of NF-*κ*B and PI3K/AKT signaling pathways were determined by Western blot. In addition, lung wet/dry (W/D) weight ratio, myeloperoxidase (MPO) activity, cell counts, and protein content were also measured.

**Results:**

According to results, AA pretreatment significantly reduced lung pathological changes, W/D ratio, MPO activity, and protein content. Additionally, AA resulted in a significant reduction in the number of total cells, neutrophils, and proinflammatory cytokines in the BALF after LPS stimulation. The subsequent study revealed that pretreatment with AA dose dependently suppressed LPS-induced activation of NF-*κ*B as well as PI3K/AKT phosphorylation.

**Conclusion:**

The results indicated that the AA had a protective effect on LPS-induced ALI in mice and could be a potential drug for ALI.

## 1. Introduction

Acute lung injury (ALI) that has cell damage of the alveolar epithelium and capillary endothelium is primarily accompanied by diffuse alveolar parenchymal damage and so on. As a result of severe ALI, acute respiratory distress syndrome (ARDS) may develop. Acute lung injury is characterized by rapid breathing, pulmonary edema, hypoxemia, and respiratory distress, which are all linked with high mortality [1]. ALI outbreak has been reported in the 2003 severe acute respiratory syndrome epidemic, as well as the current global outbreak of the corona virus disease (COVID-19). Patients with severe ALI have the symptoms of diffuse alveolar injury, lung hyaluronic membrane formation, and interstitial thickening in the lungs, which may cause pulmonary fibrosis and ARDS [2–4]. To date, effective strategies for treating ALI are lacking. NSAIDs and glucocorticoids are the main drugs used to treat ALI [5, 6], and they have serious adverse events, including upper gastrointestinal reactions, renal impairment, and arterial thrombotic events, and limited efficacy [7, 8]. Therefore, novel effective drugs that alleviate the pathological symptoms of patients with ALI should be developed. The most common precipitating factors are sepsis and severe bacterial infection. Gram-negative bacteria contain lipopolysaccharides (LPS), a component of their cell wall that causes immune and inflammatory diseases and can be used in animal models to induce ALI [9]. Therefore, a mouse ALI model was established using LPS treatment.

Aurantiamide acetate (AA) is a dipeptide derivative with a structure that resembles an endogenous peptide found in both tissues and plasma (Figure 1). It is commonly found in natural medicinal plants, such as *Baphicacanthus cusia*, *Portulaca oleracea* L., and *Clematis terniflora* DC. [10–12], exerting diverse pharmacological effects, including antiviral, antibacterial, antiparasitic, antitumor, anti-inflammatory, and antioxidant effects [10, 13–15]. The results of studies in vitro indicate that AA treatment decreases the expression of proinflammatory gene mRNA cell lines infected with influenza A virus and blocks the activation of NF-*κ*B signaling pathways, and AA effectively inhibits excessive cytokines storm and IL-6, IL-8, IP-10, TNF-*α*, and CCL5 generation in influenza A virus-infected lung epithelial cells (A549) [10]. Liu et al. [12] found that AA isolated and purified from *Clematis terniflora* DC. can inhibit the release of LPS-induced proinflammatory cytokines NO and prostaglandin E2 (PGE2) in mouse RAW264.7 cells. Besides, AA regulates MAPK and NF-*κ*B signaling pathways and exerts neuroprotection, thereby reducing LPS-induced inflammation in microglia [16].

Aside from its anti-inflammatory properties, AA appears to protect tissues and organs from damage. However, it is unclear whether AA protects against ALI. AA was examined in this study as a protective factor for lung tissue in mice undergoing LPS-induced ALI, to preliminarily explore its mechanism of action in order to discover potential therapeutic drugs for ALI treatment.

## 2. Materials and Methods

### 2.1. Reagents

AA (purity > 98%) from Chengdu Purechem-Standard Co., Ltd. (Chengdu, China) was dissolved in 0.5% sodium carboxymethyl cellulose (CMC-Na) solution. Dexamethasone acetate (Dex) was from Tianjin Tianyao Pharmaceuticals (Tianjin, China) and dissolved in normal saline with 1% DMSO. Lipopolysaccharide (LPS) was purchased from Sigma-Aldrich (St. Louis, MO, USA). The myeloperoxidase (MPO) assay kit was obtained from Nanjing Jiancheng Bioengineering Institute (Nanjing, China). TNF-*α*, IL-6, and IL-1*β* ELISA kits were purchased from BioLegend Inc. (CA, USA). All antibodies used in this study were supplied by Cell Signaling Technology Inc. (Beverly, MA).

### 2.2. Animals

We obtained adult male ICR mice from Zhejiang Laboratory Animal Centre (Hangzhou, China) that weighed 18-22 grams. During the 12-hour dark/light cycle, mice were free to eat and drink at 22-25°C. Animal experiments were performed strictly according to protocols (No. 2021R0618) approved by the Institutional Animal Care and Use Committee at the Zhejiang Laboratory Animal Center.

### 2.3. Experimental Design

Six groups of twelve ICR mice each were randomly divided: (1) the control group, (2) LPS group, (3) LPS+Dex (5 mg/kg) group (as the positive group), (4) LPS+AA (2.5 mg/kg) group, (5) LPS+AA (5 mg/kg) group, and (6) LPS+AA (10 mg/kg) group. Before LPS induction, all animals were given normal saline or drugs intragastrically for 3 days. One hour after the last gavage, inhalation of isoflurane anesthetized the mice (except for mice in control group), and 10 *μ*g/mouse LPS was infused through nasal cavity to induce ALI [17]. After 24 hours, the lung tissues of each group of mice were collected along with bronchoalveolar lavage fluid (BALF). BALF was collected via intubation of trachea and lavage (3 times with PBS, each 1.0 mL) of the lungs.

### 2.4. Lung Wet-to-Dry (W/D) Weight Ratio

Excision of right lungs of mice after euthanizing them was subsequently recorded along with their wet weight. Then, bake the lungs at 80°C for 48 hours, remove them, and measure their dry weight. To determine the extent of tissue edema, lung W/D weight ratios were calculated.

### 2.5. MPO Activity Assay

After homogenizing the mice's left lung in PBS, MPO activity was assessed using an assay kit (Nanjing Jiancheng Bioengineering Institute, Nanjing, China) according to the manufacturer's protocol.

### 2.6. Lung Histology Assay

4% neutral formaldehyde was used to fix the upper lobes of each group's left lung for 24 hours. A series of gradient concentrations of ethanol was then used to dehydrate the lung specimens, followed by xylene clearing, embedding in paraffin, and sectioning them into sections of 4 *μ*m thickness. Under light microscopy, the same location of the lung tissues is examined for pathological changes, and deparaffinization and hematoxylin and eosin (H&E) staining were done.

### 2.7. Analysis of Cell Counts in BALF

After the onset of LPS-induced lung inflammation, BALF was collected 24 hours later. After centrifugation at 3000 rpm for 10 minutes at 4°C, we collected the supernatants and frozen them at -80°C for backup. After resuspending cell pellet in 1% BSA, the total cell counts were calculated by hemocytometer, and neutrophils were counted by centrifugation, followed by Wright's stain.

### 2.8. Determination of Protein Content and Proinflammatory Cytokines

BCA protein assay kit was used to quantify protein concentrations in BALF supernatants. The expressions of IL-6, TNF-*α*, and IL-1*β* in BALF were determined according to the manufacturer's instructions using ELISA kits.

### 2.9. Western Blot Analysis

Homogenized lung tissues were washed with PBS, and then extract total protein from them using lysis buffer containing a protease inhibitor cocktail (Sigma, St. Louis, MO). Load the samples onto 10% gels and transfer onto nitrocellulose subsequently. Then, we incubated the membranes with appropriate concentrations of specific antibodies. After washing, incubate the membranes with second antibody conjugated with horseradish peroxidase. After stripping the membranes, anti-GAPDH antibody was reblotted to ensure that each lane was loaded with equal amounts of protein. The relative levels of protein expression were quantified by a densitometer (Imaging System) with respect to GAPDH. Visualization of immunoreactive bands was conducted with a phototope-horseradish peroxidase-based system (Cell Signaling Technologies, Beverly, MA), and densitometry was performed with Molecular Analyst software (Bio-Rad Laboratories, Hercules, CA).

### 2.10. Statistical Analysis

All data are expressed as means ± SD. The one-way ANOVA with or without the Tukey-Kramer multiple comparison (post hoc) tests was used in evaluating statistical differences. The least significant difference method was used in analyzing multiple comparisons with homogeneity of variance. Dunnett's T3 method was used with the heterogeneity of variance. Statistical significance was defined as *p* < 0.05 or *p* < 0.01.

## 3. Results

### 3.1. Effects of AA on Lung Histopathologic Changes

Lung pathological changes of mice in each group were assessed via H&E staining.  Figure 2 shows that the control group's lung tissues displayed normal alveolar structure and no signs of pathology. In contrast, mice in the LPS group had severely damaged lung tissue structure, with varying alveolar septa sizes, thickened and broken alveolar walls, proliferation of vascular endothelial cells, and a large amounts of neutrophil infiltration and red blood cell extravasation in the lung interstitium. However, both Dex and different doses of AA pretreatment can markedly ameliorate lung pathological damage to varying degrees, and the effect of AA was dose-dependent.

### 3.2. Effects of AA on Lung W/D Weight Ratio

The most obvious pathogenic change in ALI induced by LPS is lung edema. AA was tested 24 hours after the challenge with LPS for its effect on lung edema, and lung W/D weight ratio was determined. As exhibited in Figure 3(a), when lung W/D weight after LPS challenge is compared to those for the control group, this ratio increased significantly. AA pretreatment, however, inhibited this increased ratio in a dose-dependent fashion.

### 3.3. Effects of AA on Lung MPO Activity

Using MPO activity in lung tissues, we examined neutrophil infiltration in ALI mice induced by LPS. As illustrated in Figure 3(b), in comparison to the control group, significantly more MPO activity was observed in lung tissues in the presence of LPS. At doses of 2.5, 5, and 10 mg/kg, AA markedly inhibited this increase.

### 3.4. Effects of AA on Inflammatory Cell Count in BALF

This study was conducted to assess the amounts of total cells and neutrophils in BALF. As demonstrated in Figure 4, LPS induced a significant increase in the number of total cells and neutrophils compared to the control group. The amounts of total cells and neutrophils in LPS-stimulated cells were significantly greater than in controls. Nevertheless, in contrast with the LPS group, pretreatment with AA remarkably reduced neutrophil counts and total cells, and this change was more obvious in the LPS+AA (10 mg/kg) group.

### 3.5. Effects of AA on Protein Concentration in the BALF

As demonstrated in Figure 5(a), there was greater lung protein concentration in the LPS group than in controls. Yet, when Dex or AA was administered, lung protein concentrations were significantly reduced relative to those of the LPS group.

### 3.6. Effect of AA on Proinflammatory Cytokine Levels in the BALF

Inflammatory mediators, especially IL-6, TNF-*α*, and IL-1*β*, are crucial to the development of ALI induced by LPS. Thus, AA was tested for its ability to produce proinflammatory cytokines, TNF-*α*, IL-1*β*, and IL-6. ELISA test revealed an increase in IL-6, TNF-*α*, and IL-1*β* in BALF after LPS exposure, while AA pretreatment significantly suppressed this increase (Figures 5(b)–5(d)).

### 3.7. Effect of AA on Protein Expression of NF-*κ*B Signaling Pathway

According to research, regulation of inflammatory cytokines is carried out by NF-*κ*B. In order to elucidate AA's anti-inflammatory mechanism, we examined the NF-*κ*B signaling pathway. Compared to the control group, p-p65 expression increased and p-I*κ*B*α* was observed in the LPS group according to Western blot analysis. However, pretreatment with AA dose dependently suppressed LPS-induced activation of NF-*κ*B (Figure 6).

### 3.8. Effect of AA on Protein Expression of PI3K/AKT Signaling Pathway

Upstream of NF-*κ*B are PI3K and AKT. In this study, we assessed how AA affected the phosphorylation of PI3K and AKT in lung tissues induced by LPS. Phosphorylation levels were higher in the LPS group. On the other hand, as a result of LPS stimulation, it is dose-dependent that AA inhibits PI3K and AKT phosphorylation (Figure 7).

## 4. Discussion

Life-threatening lung diseases such as ALI and its more severe form, ARDS, are often associated with acute and severe lung inflammation. Major breakthroughs have been made in research on ALI/ARDS, but no effective drug therapy for ALI/ARDS treatment is currently available. The novel corona virus pneumonia is raging around the world, leading to severe respiratory distress syndrome [18]. Therefore, novel treatments for ALI/ARDS and severe pneumonia (such as COVID-19) are in high demand on the market.

Plant-derived natural products have many active compounds with novel structures, multitargeting capability, high activity, and low side effects, showing potential as drugs and important sources of anti-inflammatory agents [19, 20]. Microsomal prostaglandin E synthase-1 (mPGES-1) is an enzyme that is crucial for the production of PGE2 during inflammation, and anti-inflammatory drugs could be developed targeting this target [21]. Chen et al. [22] screened the potential inhibitors of mPGES-1 from the TCM Database@Taiwan. They found that AA conforms to the pharmacophore and quantitative structure–activity relationship model and has a high docking score and binding stability with mPGES-1. The biological activity of AA was predicted using multiple linear regression and support vector machine, which corroborated its anti-inflammatory activity. AA has an inhibitory effect on superoxide formation and histamine release and inhibits the expression of LPS-induced proinflammatory cytokines (TNF-*α* and IL-2) [23]. Additionally, it has selective inhibitory effect against superoxide anions generation and overreleased elastase by fMLP/CB-induced human neutrophils and overreleased elastase [24]. Therefore, AA is a candidate compound for anti-inflammatory drug development.

In this study, neutrophils in BALF increased significantly as a result of LPS exposure, whereas AA pretreatment significantly decreased the level of neutrophils. Neutrophils contain a significant quantity of MPO in their cytoplasmic granules, and thus, its level and activity in tissues represent the function and activity of neutrophils [25]. We found that after exposure to LPS, MPO activity was remarkably enhanced in lung tissues but significantly reduced after AA pretreatment. Histopathological results further confirmed that AA could inhibit neutrophil infiltration in lung tissues.

LPS triggers the release of several inflammation-related cytokines and chemokines [26]. Activated TNF-*α*, IL-1*β*, and IL-6 do not only initiate but also amplify and prolong ALI's inflammatory response [27]. An inflammatory response starts with TNF-*α* as its initial and most important mediator. It is mainly produced by activated monocytes or macrophages and causes an inflammatory cascade response that damages the endothelial cells of the vascular system while also inducing the alveolar epithelial system to release other cytokines, IL-6, for example [28]. Following LPS exposure, IL-6, IL-1*β*, and TNF-*α* were significantly elevated in BALF, but the levels were markedly reduced after AA pretreatment. As a symptom of inflammation, an indicator of pulmonary edema is the lung W/D weight ratio. Based on three results, AA reduced the lung W/D ratio and alleviated pulmonary edema symptoms, suggesting ALI induced by LPS is protected against by it.

NF-*κ*B is a transcription factor involved in producing inflammatory cytokines, which is essential for the development of inflammatory diseases like ALI, chronic obstructive pulmonary disease, and pulmonary fibrosis. It is possible to alleviate lung inflammation by inhibiting NF-*κ*B activation [10, 29, 30]. Activation of PI3K/AKT can promote the translocation of NF-*κ*B, as well as its transcriptional activity, thus directly affecting inflammatory cytokine expression [31]. Acute pancreatitis-related lung injury is caused by the PI3K/AKT/NF-*κ*B signaling pathway, which activate inflammatory cytokines [32]. In this study, we measured the expression of NF-*κ*B p65, NF-*κ*B p-p65, I*κ*B*α*, p-I*κ*B*α*, PI3K, p-PI3K, AKT, and p-AKT in lung tissues by Western blot. The p-I*κ*B*α*/I*κ*B*α*, p-p65/p65, p-PI3K/PI3K, and AKT/p-AKT ratios in the LPS group significantly increased. AA pretreatment led to a dose-dependent reduction in these levels compared with the LPS group. It is believed that NF-*κ*B dimers bind to inhibitory protein I*κ*B*α* under normal conditions and are inactive in the cytoplasm. The dissociation of NF-*κ*B p65 from I*κ*B*α* by LPS leads to its translocation to the nucleus and inflammatory cytokine genes by which transcription is controlled [33]. Therefore, LPS exposure can lead to the degradation of I*κ*B*α*, which can be blocked by AA pretreatment. Taken together, these data suggest that the alleviating effect of AA on LPS-induced lung inflammation may be partly related to the inhibition of NF-*κ*B activation as well as PI3K/AKT phosphorylation.

Collectively, this study revealed the potent protective effect of AA against LPS-induced ALI, which may be linked to its anti-inflammatory activities. It appears that AA is a promising treatment for ALI. However, further studies are recommended for better elucidation of the underlying molecular mechanisms of AA.

## Figures and Tables

**Figure 1:** Chemical structure of AA.

**Figure 2:** Effects of AA on histopathological changes in lung tissues in LPS-induced ALI mice. Representative histological changes of lung obtained from mice of different groups (magnification ×200).

**Figure 3:** Effects of AA on lung W/D ratio and MPO activity in ALI mice. Data are expressed as the mean ± SD (*n* = 6). ^#^*p* < 0.05 and ^##^*p* < 0.01 vs. control group. ^∗^*p* < 0.05 and ^∗∗^*p* < 0.01 vs. LPS group.

**Figure 4:** Effects of AA on inflammatory cell count. (a) Total cell count and (b) neutrophil count in BALF. Data are expressed as the mean ± SD (*n* = 6). ^#^*p* < 0.05 and ^##^*p* < 0.01 vs. control group. ^∗^*p* < 0.05 and ^∗∗^*p* < 0.01 vs. LPS group.

**Figure 5:** Effects of AA on levels of inflammatory factors in BALF. (a) Total protein concentration, (b) IL-6 concentration, (c) IL-1*β* concentration, and (d) TNF-*α* concentration in BALF in each group. Data are expressed as the mean ± SD (*n* = 6). ^#^*p* < 0.05 and ^##^*p* < 0.01 vs. control group. ^∗^*p* < 0.05 and ^∗∗^*p* < 0.01 vs. LPS group.

**Figure 6:** AA pretreatment inhibits LPS-induced NF-*κ*B activation. (a) Western blot analysis of p-I*κ*B*α*, I*κ*B*α*, p-p65, and p65 expressions in lung tissue. GAPDH was used as the loading control. (b–c) Quantitative analysis of (a). Data are presented as the mean ± SD, repeated for three times. ^#^*p* < 0.05 and ^##^*p* < 0.01 vs. control group. ^∗^*p* < 0.05 and ^∗∗^*p* < 0.01 vs. LPS group.

**Figure 7:** AA pretreatment inhibits the activation of PI3K/AKT signaling in LPS-induced ALI. (a) Western blot analysis of p-PI3K, PI3K, p-AKT, and AKT expressions in lung tissue. GAPDH was used as the loading control. (b–c) Quantitative analysis of (a). Data are presented as the mean ± SD, repeated for three times. ^#^*p* < 0.05 and ^##^*p* < 0.01 vs. control group. ^∗^*p* < 0.05 and ^∗∗^*p* < 0.01 vs. LPS group.

## Data Availability

All data generated or analyzed during this study are included in this article.

## References

[1] Mowery N. T., Terzian W. T. H., Nelson A. C. (2020). Acute lung injury. *Current Problems in Surgery*.

[2] He L., Ding Y., Zhang Q. (2006). Expression of elevated levels of pro-inflammatory cytokines in SARS-CoV-infected ACE2+ cells in SARS patients: relation to the acute lung injury and pathogenesis of SARS. *The Journal of Pathology*.

[3] Camporota L., Cronin J. N., Busana M., Gattinoni L., Formenti F. (2022). Pathophysiology of coronavirus-19 disease acute lung injury. *Current Opinion in Critical Care*.

[4] Li L., Huang Q., Wang D. C., Ingbar D. H., Wang X. (2020). Acute lung injury in patients with COVID-19 infection. *Clinical and Translational Medicine*.

[5] Bruce E., Barlow-Pay F., Short R. (2020). Prior routine use of non-steroidal anti-inflammatory drugs (NSAIDs) and important outcomes in hospitalised patients with COVID-19. *Journal of Clinical Medicine*.

[6] Tomazini B. M., Maia I. S., Cavalcanti A. B. (2020). Effect of dexamethasone on days alive and ventilator-free in patients with moderate or severe acute respiratory distress syndrome and COVID-19: the CoDEX randomized clinical trial. *Journal of the American Medical Association*.

[7] Cumhur Cure M., Kucuk A., Cure E. (2020). NSAIDs may increase the risk of thrombosis and acute renal failure in patients with COVID-19 infection. *Thérapie*.

[8] Lu S., Zhou Q., Huang L. (2020). Effectiveness and safety of glucocorticoids to treat COVID-19: a rapid review and meta-analysis. *Annals of Translational Medicine*.

[9] Chen H., Bai C., Wang X. (2010). The value of the lipopolysaccharide-induced acute lung injury model in respiratory medicine. *Expert Review of Respiratory Medicine*.

[10] Zhou B., Yang Z., Feng Q. (2017). Aurantiamide acetate from Baphicacanthus cusia root exhibits anti-inflammatory and anti-viral effects via inhibition of the NF-*κ*B signaling pathway in influenza A virus-infected cells. *Journal of Ethnopharmacology*.

[11] Chen L., Liu Y., Jia D. (2016). Pharmacokinetics and biodistribution of aurantiamide and aurantiamide acetate in rats after oral administration of Portulaca oleracea L. extracts. *Journal of Agricultural And Food Chemistry*.

[12] Liu X. B., Yang B. X., Zhang L., Lu Y. Z., Gong M. H., Tian J. K. (2015). An in vivo and in vitro assessment of the anti-inflammatory, antinociceptive, and immunomodulatory activities of Clematis terniflora DC. extract, participation of aurantiamide acetate. *Journal of Ethnopharmacology*.

[13] Tamokou J. D. D., Simo Mpetga D. J., Keilah Lunga P., Tene M., Tane P., Kuiate J. R. (2012). Antioxidant and antimicrobial activities of ethyl acetate extract, fractions and compounds from stem bark of Albizia adianthifolia (Mimosoideae). *BMC Complementary and Alternative Medicine*.

[14] Yang Y., Zhang L. H., Yang B. X., Tian J. K., Zhang L. (2015). Aurantiamide acetate suppresses the growth of malignant gliomas in vitro and in vivo by inhibiting autophagic flux. *Journal of Cellular and Molecular Medicine*.

[15] Igoli N. P., Clements C. J., Singla R. K., Igoli J., Uche N., Gray A. (2014). Antitrypanosomal activity & docking studies of components of Crateva adansonii DC leaves: novel multifunctional scaffolds. *Current Topics in Medicinal Chemistry*.

[16] Yoon C. S., Kim D. C., Lee D. S. (2014). Anti-neuroinflammatory effect of aurantiamide acetate from the marine fungus Aspergillus sp. SF-5921: inhibition of NF-*κ*B and MAPK pathways in lipopolysaccharide-induced mouse BV2 microglial cells. *International Immunopharmacology*.

[17] Zhu H., Wang Y., Sun J., Fan C., Wan J. (2020). Tomentosin inhibits lipopolysaccharide-induced acute lung injury and inflammatory response by suppression of the NF-*κ*B pathway in a mouse model of sepsis. *Journal of Environmental Pathology, Toxicology and Oncology*.

[18] Batah S. S., Fabro A. T. (2021). Pulmonary pathology of ARDS in COVID-19: a pathological review for clinicians. *Respiratory Medicine*.

[19] He Y. Q., Zhou C. C., Yu L. Y. (2021). Natural product derived phytochemicals in managing acute lung injury by multiple mechanisms. *Pharmacological Research*.

[20] Ding C., Chen H., Liang B., Jiao M., Liang G., Zhang A. (2019). Biomimetic synthesis of the natural product salviadione and its hybrids: discovery of tissue-specific anti-inflammatory agents for acute lung injury. *Chemical Science*.

[21] Ding K., Zhou Z., Hou S. (2018). Structure-based discovery of mPGES-1 inhibitors suitable for preclinical testing in wild-type mice as a new generation of anti-inflammatory drugs. *Scientific Reports*.

[22] Chen K. C., Sun M. F., Yang S. C. (2011). Investigation into potent inflammation inhibitors from traditional Chinese medicine. *Chemical Biology & Drug Design*.

[23] Ng T. B., Liu F., Lu Y., Cheng C. H., Wang Z. (2003). Antioxidant activity of compounds from the medicinal herb Aster tataricus. *Comp Biochem Physiol C Toxicol Pharmacol*.

[24] Yen C. T., Hwang T. L., Wu Y. C., Hsieh P. W. (2009). Design and synthesis of new N-(fluorenyl-9-methoxycarbonyl) (Fmoc)-dipeptides as anti-inflammatory agents. *European Journal of Medicinal Chemistry*.

[25] Flores-Huerta N., Pacheco-Yépez J., Sánchez-Monroy V. (2020). The MPO system participates actively in the formation of an oxidative environment produced by neutrophils and activates the antioxidant mechanism of Naegleria fowleri. *Journal of Leukocyte Biology*.

[26] Tirunavalli S. K., Gourishetti K., Kotipalli R. S. S. (2021). Dehydrozingerone ameliorates lipopolysaccharide induced acute respiratory distress syndrome by inhibiting cytokine storm, oxidative stress via modulating the MAPK/NF-*κ*B pathway. *Phytomedicine*.

[27] Jiang W. Y., Ren J., Zhang X. H. (2020). CircC3P1 attenuated pro-inflammatory cytokine production and cell apoptosis in acute lung injury induced by sepsis through modulating miR-21. *Journal of Cellular and Molecular Medicine*.

[28] Chen D., Chen C., Xiao X., Huang Z., Huang X., Yao W. (2021). TNF-*α* induces neutrophil apoptosis delay and promotes intestinal ischemia- reperfusion-induced lung injury through activating JNK/FoxO3a pathway. *Oxidative Medicine and Cellular Longevity*.

[29] Xiong Y., Cui X., Zhou Y. (2021). Dehydrocostus lactone inhibits BLM-induced pulmonary fibrosis and inflammation in mice via the JNK and p38 MAPK-mediated NF-*κ*B signaling pathways. *International Immunopharmacology*.

[30] Liu Y., Huang Z. Z., Min L., Li Z. F., Chen K. (2021). The BRD4 inhibitor JQ1 protects against chronic obstructive pulmonary disease in mice by suppressing NF-*κ*B activation. *Histology and Histopathology*.

[31] Urbani C., Mattiello A., Ferri G. (2021). PCB153 reduces apoptosis in primary cultures of murine pituitary cells through the activation of NF-*κ*B mediated by PI3K/Akt. *Molecular and Cellular Endocrinology*.

[32] Jin Y., Liu L., Chen B. (2017). Involvement of the PI3K/Akt/NF-*κ*B signaling pathway in the attenuation of severe acute pancreatitis-associated acute lung injury by Sedum sarmentosum Bunge extract. *BioMed Research International*.

[33] Chen K. L., Li L., Li C. M. (2019). SIRT7 regulates lipopolysaccharide-induced inflammatory injury by suppressing the NF-*κ*B signaling pathway. *Oxidative Medicine and Cellular Longevity*.

